The article "Exploration of inhibitory mechanisms of curcumin in lung cancer metastasis using a miRNA- transcription factor-target gene network" was retracted in 2017. Reason: errors in the materials.

# Exploration of inhibitory mechanisms of curcumin in lung cancer metastasis using a miRNA- transcription factor-target gene network

**DOI:** 10.1371/journal.pone.0172470

**Published:** 2017-02-23

**Authors:** De-min Jiao, Li Yan, Li-shan Wang, Hui-zhen Hu, Xia-li Tang, Jun Chen, Jian Wang, You Li, Qing-yong Chen

**Affiliations:** 1 Department of Respiratory Disease, The 117th Hospital of PLA, Hangzhou, Zhejiang, P.R. China; 2 Department of Oncology, The 117th Hospital of PLA, Hangzhou, Zhejiang, P.R. China; 3 Bio-X Institutes, Key Laboratory for the Genetics of Developmental and Neuropsychiatric Disorders (Ministry of Education), Shanghai Jiao Tong University, Shanghai, P.R. China; Baylor University Medical Center, UNITED STATES

## Abstract

The present study was aimed to unravel the inhibitory mechanisms of curcumin for lung cancer metastasis via constructing a miRNA-transcription factor (TF)-target gene network. Differentially expressed miRNAs between human high-metastatic non-small cell lung cancer 95D cells treated with and without curcumin were identified using a TaqMan human miRNA array followed by real-time PCR, out of which, the top 6 miRNAs (miR-302b-3p, miR-335-5p, miR-338-3p, miR-34c-5p, miR-29c-3p and miR-34a-35p) with more verified target genes and TFs than other miRNAs as confirmed by a literature review were selected for further analysis. The miRecords database was utilized to predict the target genes of these 6 miRNAs, TFs of which were identified based on the TRANSFAC database. The findings of the above procedure were used to construct a miRNA-TF-target gene network, among which miR-34a-5p, miR-34c-5p and miR-302b-3p seemed to regulate CCND1, WNT1 and MYC to be involved in Wnt signaling pathway through the LEF1 transcription factor. Therefore, we suggest miR-34a-5p/miR-34c-5p/miR-302b-3p —LEF1—CCND1/WNT1/MYC axis may be a crucial mechanism in inhibition of lung cancer metastasis by curcumin.

## Introduction

Lung cancer, predominantly non-small-cell lung cancer (NSCLC), is the most common cause of cancer mortality in the United States, with an estimated 158,080 cancer deaths occurred in 2016 [1]. Metastatic progression is the main factor to result in the poor prognosis of patients [2]. Exploration of strategies to inhibit metastasis has justifiably attracted enormous attention in clinic.

Curcumin, a natural polyphenol derived from turmeric (Curcuma longa), is one of the most widely investigated compounds recently due to its protective property against cancer [3, 4]. Curcumin may suppress the invasion and metastasis of lung cancer cells by downregulating the expression of matrix metalloproteinases, which can be medicated by protein kinase Cα (PKCα) / NADPH oxidase-2 (Nox-2) / reactive oxygen species (ROS) / activating transcription factor-2 (ATF-2) [5] or glucose transporter 1 (GLUT1) / membrane type 1-MMP (MT1-MMP) [6]. Furthermore, evidence is also provided to indicate the inactivation of Wnt/β-catenin pathway in the therapeutic process of curcumin [7]. However, the inhibitory mechanisms of curcumin in lung cancer metastasis remain under investigation.

The article "Exploration of inhibitory mechanisms of curcumin in lung cancer metastasis using a miRNA- transcription factor-target gene network" was retracted in 2017. Reason: errors in the materials.

A consensus has been reached that gene expression can be regulated by microRNAs (miRNAs) via binding to its 3′ untranslated regions [8]. Thus, we hypothesize curcumin may regulate its target gene expression by controlling miRNAs, thus affecting lung cancer metastasis. This hypothesis has been demonstrated by recent studies as follows: Jin *et al*. report that curcumin may inhibit proliferation and promote apoptosis of NSCLC cells via upregulation of miR-192-5p followed by inhibition of PI3K/Akt pathway [9]. The study of Ye *et al*. highlights the pro-apoptotic effects of curcumin depend on induction of miR-192-5p/215 followed by targeting X-linked inhibitor of apoptosis (XIAP) gene [10]. Nevertheless, the research on the miRNAs that were changed after curcumin treatment remains limited and rare studies focused on miRNAs associated with lung cancer metastasis.

The goal of this study was to screen crucial miRNAs that were differentially expressed in high-metastatic NSCLC cells undergoing curcumin treatment or not by the use of a miRNA microarray analysis. The target genes of miRNAs and their function were also predicted. The findings of our study may further unearth the inhibitory mechanisms of curcumin in lung cancer metastasis and provide new therapeutic targets for lung cancer.

## Materials and methods

### Reagents and cell culture

Curcumin was purchased from Sigma Chemical Company (St Louis, MO, USA). A 100 mM stock solution of curcumin was prepared in dimethyl sulfoxide (Sigma, St Louis, MO, USA) and stored at—20°C.

Human high-metastatic NSCLC 95D cell line was obtained from the Cell Bank at the Chinese Academy of Sciences (Shanghai, China). The cells were cultured in RPMI 1640 medium supplemented with 10% fetal bovine serum (Hyclone, Logan, Utah, USA), 100 units/mL penicillin and streptomycin at 37°C in 5% CO_2_.

### 3-(4,5-dimethylthiazol-2-yl)-2,5-diphenyl tetrazolium bromide (MTT) assay

Cell viability was measured by MTT assay following the instructions of the manufacturer. Briefly, cells were seeded on 96-well plates (Corning Incorporation, Corning, NY, USA) at a density of 5 × 10^3^ cells/well and grown overnight. The absorption was determined at 570 nm using an automated plate reader (Shenzhen Procan Electronics Incorporation, Rayto, Shenzhen, China). Each experimental condition was performed in triplicate.

The article "Exploration of inhibitory mechanisms of curcumin in lung cancer metastasis using a miRNA- transcription factor-target gene network" was retracted in 2017. Reason: errors in the materials.

### Wound healing assay

The 95D cells were seeded into a six-well plate and grown to confluence. Wound was created by scraping confluent cell monolayers with a 10 μL pipette tip. The cells treated with different concentrations of curcumin (0 μM, 10 μM or 20 μM) were allowed to migrate for 24 h. At 0 h and 24 h after scratching, images were taken under an inverted microscope (Olympus IX71, Olympus, China, × 40). The gap distance was measured by the Image J software (National Institute of Mental Health, Bethesda, MD, USA). Migration rate = gap distance (24 h) / gap distance (0 h).

### Cell invasion assay

Invasion assay was carried out using modified matrigel boyden chambers which consisted of a 24-well Millicell (Millipore Corporation, Shanghai, China) membrane filter (8 μm pore size) as described previously [11]. Matrigel was diluted to 200 μg/mL with cold distilled water and applied to the top side of filter. Briefly, cells were trypsinized and resuspended in serum-free medium. A total of 10^5^ cells were added to the upper chamber of each well. The bottom chambers were filled with 500 μL RPMI 1640 medium supplemented with 10% FBS and different concentrations of curcumin (10 or 20 μM). The chamber was incubated for 24 h at 37°C. At the end of incubation, cells located on the upper surface of the membrane were carefully removed with a cotton swab. Cells invading through the matrigel to the lower surface of the membrane were fixed with methanol and stained with 0.5% crystal violet. The invading cells on the lower surface of the membrane filter were counted under a light microscope (Puzhe ThotoElectric Company, Leica, Shenzhen, China). The data presented were the average number of cells attached to the bottom surface from five random fields. Each experiment was carried out in triplicate.

### miRNAs assay

Differentially expressed miRNAs between 95D cell samples treated with or without 10 μM curcumin, were identified based on the platform: TaqMan Array Human MicroRNA A+B Card Set v3 (Life Technologies, Carlsbad, California, USA) and real-time analysis of 770 human miRNAs (Sanger miRBase v18) using a 7900HT RT-PCR System (Life Technologies, Carlsbad, California, USA), with fold change (FC) > 2.0 or < 0.05 and p-value < 0.05 as the cutoff point.

Out of these identified differentially expressed miRNAs, the top six miRNAs with more verified target genes and TFs than other miRNAs in lung cancer review literatures were selected for further analysis. Subsequently, the experimentally verified target genes of the 6 miRNAs were identified using miRecords database (http://miRecords.umn.edu/miRecords) which is an integrated resource containing 1135 validated miRNA-target interactions in seven animal species [12]. Furthermore, TFs were screened out from the experimentally verified target genes according to the TRANSFAC database (http://www.gene-regulation.com/cgi-bin/pub/databases/transfac/) [13].

The article "Exploration of inhibitory mechanisms of curcumin in lung cancer metastasis using a miRNA- transcription factor-target gene network" was retracted in 2017. Reason: errors in the materials.

In addition, all potential target genes of the 6 miRNAs with biological complexity (BC) > 6 were also predicted according to miRecords database to further analyze how the 6 selected miRNAs played roles in the inhibition of NSCLC by curcumin. Similarly, TFs were screened from the predicted target genes and the targets genes of the screened TFs were determined based on the TRANSFAC database. Eventually, a miRNA-TF-target gene network was constructed using The Search Tool for the Retrieval of Interacting Genes (STRING) [14] and visualized by Cytoscape software (http://www.cytoscape.org/) [15].

### Gene ontology and Kyoto encyclopedia of genes and genomes pathway enrichment analysis

Gene ontology (GO) and Kyoto encyclopedia of genes and genomes (KEGG) pathway enrichment analyses were performed for the experimentally verified target genes of the selected 6 miRNAs and network genes using The Database for Annotation, Visualization and Integrated Discovery (DAVID) tool (http://david.abcc.ncifcrf.gov). Bonferroni adjusted p-value < 0.05 and false discovery rate (FDR) < 0.05 were chosen as cut-off criterion for GO and KEGG analyses.

### Protein-protein interaction network construction

A protein-protein interactions (PPI) network was built with the target genes of the 6 miRNAs using STRING software [16] to analyze the interactions between these target genes. The PPIs with scores > 0.4 was included in the PPI network.

## Results

### Effect of curcumin on 95D cell viability

Cell viability of the control group (0 μM curcumin) was designated as 100% in our study. As shown in Fig 1, cell viability was insignificantly decreased in response to 10 μM curcumin treatment for 24 h. However, it was decreased to 49% in cells exposed to 20 μM curcumin compared with the control group (p < 0.01). The viability of 95D cells on exposure to 40 μM curcumin was further reduced.

**Fig 1:** Curcumin inhibits 95D cell proliferation. Columns represent the mean values from three different duplicates and bars stand for standard error. **, p < 0.01 compared with 0 μM curcumin group.

### Effect of curcumin on 95D cell migration and invasion

Based on the cell viability results, the concentrations of 10 μM and 20 μM were chosen to determine the effect of curcumin on 95D cells migration and invasion. The results indicated both 10 μM and 20 μM could significantly repress 95D cells migration (Fig 2A and 2B, p < 0.01) and invasion (Fig 2C and 2D, p < 0.01). Notably, 10 μM curcumin inhibited cell migration and invasion obviously, but did not result in a significant reduction in cell viability, suggesting that 10 μM would be a suitable concentration to unravel the molecular mechanisms underlying the anti-tumor metastasis action of curcumin.

The article "Exploration of inhibitory mechanisms of curcumin in lung cancer metastasis using a miRNA- transcription factor-target gene network" was retracted in 2017. Reason: errors in the materials.

**Fig 2:** Curcumin inhibits 95D cell migration and invasion. (A) 95D confluent monolayer cells are scratched with a pipette tip and then treated with 10 μM or 20 μM curcumin. Representative images show the inhibitory effect of curcumin on 95D cell at 24 h. (B) The gap distance is quantitatively evaluated using the Image J software. (C) The invasion ability of 95D cell is determined by invasion assay. Cells in low surface of the Boyden chamber are stained and photographed under a light microscope at × 100 magnification. (D) The invading cells are quantified by counting the number of stained cells under a light microscope at × 200 magnification. Columns, mean from three different experiments with 3 duplicates; *, p < 0.05; **, p < 0.01 compared with 0 μM curcumin group.

### Identification of crucial differentially expressed miRNAs and their experimentally validated target genes and TFs

Totally, 36 differentially expressed miRNAs were identified between 95D cells treated with and without curcumin (FC > 2.0 or < 0.05 and p < 0.05, Table 1). Further, 6 miRNAs (miR-302b-3p, miR-335-5p, miR-338-3p, miR-34c-5p, miR-29c-3p and miR-34a-35p) with more verified target genes and TFs than others in lung cancer review literatures were screened, suggesting these 6 miRNAs might play critical roles in the suppression of lung cancer metastasis by curcumin. Based on the miRecords database, 39 experimentally verified target genes of these 6 miRNAs were identified (Table 2), of which three genes were recognized as TFs based on TRANSFAC database, including E2F transcription factor 3 (E2F3), v-myb avian myelocytomatosis viral oncogene homolog (MYB) and v-myc avian myelocytomatosis viral oncogene homolog (MYC).

**Table 1:** The 36 differentially expressed miRNAs between curcumin-treated group and control group.

miRBase-human-18th	Target sequence	Fold change
hsa-miR-330-5p	UCUCUGGGCCUGUGUCUUAGGC	142.34
hsa-miR-331-5p	CUAGGUAUGGUCCCAGGGAUCC	70.74
hsa-miR-1276	UAAAGAGCCCUGUGGAGACA	45.97
hsa-miR-544a	AUUCUGCAUUUUUAGCAAGUUC	15.27
hsa-miR-29c-5p	UGACCGAUUUCUCCUGGUGUUC	10.96
hsa-miR-335-5p	UCAAGAGCAAUAACGAAAAAUGU	10.09
hsa-miR-296-3p	GAGGGUUGGGUGGAGGCUCUCC	8.59
hsa-miR-34a-5p	UGGCAGUGUCUUAGCUGGUUGU	7.26
hsa-miR-26a-1-3p	CCUAUUCUUGGUUACUUGCACG	6.63
hsa-miR-190a	UGAUAUGUUUGAUAUAUUAGGU	4.66
hsa-miR-362-3p	AACACACCUAUUCAAGGAUUCA	4.52
hsa-let-7f-2-3p	CUAUACAGUCUACUGUCUUUCC	4.26
hsa-miR-302b-3p	UAAGUGCUUCCAUGUUUUAGUAG	3.34
hsa-miR-338-3p	UCCAGCAUCAGUGAUUUUGUUG	2.86
hsa-miR-455-3p	GCAGUCCAUGGGCAUAUACAC	2.17
hsa-miR-29c-3p	UAGCACCAUUUGAAAUCGGUUA	0.49
hsa-miR-154-3p	AAUCAUACACGGUUGACCUAUU	0.48
hsa-miR-21-3p	CAACACCAGUCGAUGGGCUGU	0.45
hsa-miR-377-5p	AGAGGUUGCCCUUGGUGAAUUC	0.43
hsa-miR-34c-5p	AGGCAGUGUAGUUAGCUGAUUGC	0.37
hsa-miR-1257	AGUGAAUGAUGGGUUCUGACC	0.31
hsa-miR-744-3p	CUGUUGCCACUAACCUCAACCU	0.31
hsa-miR-502-5p	AUCCUUGCUAUCUGGGUGCUA	0.27
hsa-miR-33a-3p	CAAUGUUUCCACAGUGCAUCAC	0.23
hsa-miR-424-3p	CAAAACGUGAGGCGCUGCUAU	0.21
hsa-miR-92a-1-5p	AGGUUGGGAUCGGUUGCAAUGCU	0.17
hsa-miR-10b-3p	ACAGAUUCGAUUCUAGGGGAAU	0.15
hsa-miR-769-3p	CUGGGAUCUCCGGGGUCUUGGUU	0.06
hsa-miR-1179	AAGCAUUCUUUCAUUGGUUGG	0.05
hsa-miR-516a-3p	UGCUUCCUUUCAGAGGGU	0.05
hsa-miR-148a-5p	AAAGUUCUGAGACACUCCGACU	0.05
hsa-miR-604	AGGCUGCGGAAUUCAGGAC	0.04
hsa-miR-499a-5p	UUAAGACUUGCAGUGAUGUUU	0.04
hsa-miR-1262	AUGGGUGAAUUUGUAGAAGGAU	0.04
hsa-let-7a-3p	CUAUACAAUCUACUGUCUUUC	0.03
hsa-miR-25-5p	AGGCGGAGACUUGGGCAAUUG	0.005

The article "Exploration of inhibitory mechanisms of curcumin in lung cancer metastasis using a miRNA- transcription factor-target gene network" was retracted in 2017. Reason: errors in the materials.

**Table 2:** The verified target genes of the 6 miRNAs.

miRNA	Genes count	Validated target genes
hsa-miR-302b-3p	3	CCND1, LEFTY1, LEFTY2
hsa-miR-335-5p	0	---------
hsa-miR-338-3p	1	UBE2Q1
hsa-miR-34c-5p	1	MYC
hsa-miR-29c-5p	14	LAMC1, DNMT3A, DNMT3B, COL3A1, COL4A1, COL3A1, COL15A1, TDG, FUSIP1, COL1A1, COL1A2, COL4A2, FBN1, FIK3R1, CDC42,
hsa-miR-34a-5p	20	DLL1, NOTCH1, BCL2, E2F3, CDK6, VEGFA, MYCN, NOTCH2, SIRT1, CCND1, MYB, MYC, Notch-1, JAG1, MET, MAP2K1, AXIN2, WNT1, CD44, Axl, EphA5

Note: 0 and --------- represent none of the validated target genes have been discovered.

Function enrichment analysis showed that these 39 verified target genes were mainly involved in 10 significant GO terms (Table 3) and 4 significant KEGG pathways (Table 4). The most significant term was regulation of cell proliferation (Bonferroni adjusted p-value = 8.66E^-05^, FDR = 1.34E^-04^), with 13 genes enriched, such as E2F3, MYC, NOTCH1, NOTCH2, cyclin-dependent kinase 6 (CDK6), B-cell lymphoma 2 (BCL2) and cyclin-D1 (CCND1). Besides, the terms of epithelium, epidermis and ectoderm development may be associated with cell migration, with NOTCH1, mitogen-activated protein 2 kinase 1 (MAP2K1) and BCL2 enriched. The identified KEGG pathways were all related with cancer development (pathways in cancer, focal adhesion, small cell lung cancer and pancreatic cancer) and migration (focal adhesion), with CCND1 enriched in all pathways.

**Table 3:** Gene Ontology (GO) term enrichment analysis.

	Category ID	Term	Genes	Bonferroni adjusted p-value	FDR
A	GO:0042127	Regulation of cell proliferation	E2F3, CDK6, JAG1, SIRT1, LEFTY1, MYCN, NOTCH2, NOTCH1, CCND1, BCL2, VEGFA, AXIN2, MYC	8.66E-05	1.34E-04
	GO:0001709	Cell fate determination	CDC42, WNT1, NOTCH2, DLL1, JAG1	1.23 E-03	1.90E-03
	GO:0045165	Cell fate commitment	CDC42, WNT1, NOTCH2, NOTCH1, BCL2, DLL1, JAG1	1.90 E-03	2.94E-03
	GO:0060429	Epithelium development	NOTCH2, NOTCH1, COL4A1, CD44, MAP2K1, BCL2, VEGFA, JAG1	3.49E-03	5.41E-03
	GO:0008544	Epidermis development	NOTCH1, MAP2K1, BCL2, COL3A1, COL1A2, COL1A1	8.14E-03	1.27E-02
	GO:0007398	Ectoderm development	NOTCH1, MAP2K1, BCL2, COL3A1, COL1A2, COL1A1	1.22E-02	1.91E-02
	GO:0045596	Negative regulation of cell differentiation	CCND1, NOTCH1, DLL1, CDK6, JAG1, AXIN2, SIRT1	2.05E-02	3.20E-02
	GO:0030182	Neuron differentiation	CDC42, WNT1, NOTCH1, CD44, MAP2K1, BCL2, VEGFA, DLL1, JAG1	2.39E-02	3.74E-02
	GO:0048730	Epidermis morphogenesis	NOTCH1, BCL2, COL1A2, COL1A1	2.78E-02	4.36E-02
	GO:0048729	Tissue morphogenesis	NOTCH2, NOTCH1, CD44, BCL2, COL1A2, JAG1, COL1A1	3.00E-02	4.70E-02
B	GO:0030097	Hemopoiesis	LMO2, LYN, TP53, DLL1, RAG2, RUNX1, TCF3, ADA, CTNNB1, CD1D, TIMP1	3.67E-05	5.11E-05
	GO:0016055	Wnt receptor signaling pathway	WNT1, CCND1, MITF, TLE4, LEF1, TLE1, MARK4, TCF7L1, CTNNB1	6.74E-05	9.39E-05
	GO:0048534	Hemopoietic or lymphoid organ development	LMO2, LYN, TP53, DLL1, RAG2, RUNX1, TCF3, ADA, CTNNB1, CD1D, TIMP1	9.14E-05	1.27E-04
	GO:0002520	Immune system development	LMO2, LYN, TP53, DLL1, RAG2, RUNX1, TCF3, ADA, CTNNB1, CD1D, TIMP1	1.60E-04	2.22E-04
	GO:0042127	Regulation of cell proliferation	ODC1, E2F3, LYN, BECN1, MITF, TP53, MMP7, MARK4, ADA, TIMP1, CTNNB1, CCND1, IFNB1, TCF3, MYC, PLAU	4.00E-04	5.56E-04
	GO:0045893	Positive regulation of transcription, DNA-dependent	WNT1, E2F3, MITF, TP53, LEF1, RUNX1, ALX4, TCF3, MYC, TCF7L1, TP73, CTNNB1	3.16E-03	4.41E-03
	GO:0051254	Positive regulation of RNA metabolic process	WNT1, E2F3, MITF, TP53, LEF1, RUNX1, ALX4, TCF3, MYC, TCF7L1, TP73, CTNNB1	3.43E-03	4.78E-03
	GO:0045941	Positive regulation of transcription	WNT1, E2F3, MITF, TP53, LEF1, RUNX1, ALX4, TCF3, MYC, TCF7L1, TP73, CTNNB1	1.55E-02	2.17E-02
	GO:0010628	Positive regulation of gene expression	WNT1, E2F3, MITF, TP53, LEF1, RUNX1, ALX4, TCF3, MYC, TCF7L1, TP73, CTNNB1	2.04E-02	2.89E-02
	GO:0045165	Cell fate commitment	WNT1, MITF, TP53, DLL1, RAG2, TCF3, CTNNB1	2.31E-02	3.26E-02
	GO:0009952	Anterior/posterior pattern formation	WNT1, HOXC13, LEF1, DLL1, ALX4, TCF7L1, CTNNB1	2.41E-02	3.39E-02
	GO:0006357	Regulation of transcription from RNA polymerase II promoter	ELF2, MITF, TP53, LEF1, TLE1, SNAI2, TCF7L1, CTNNB1, IRF2, ALX4, RUNX1, MYC, TCF3	3.12E-02	4.42E-02

FDR, false discovery rate; A, pathway enrichment analysis of the verified target genes of miRNAs; B, pathway enrichment analysis of genes in the miRNAs-transcription factors-target genes network.

The article "Exploration of inhibitory mechanisms of curcumin in lung cancer metastasis using a miRNA- transcription factor-target gene network" was retracted in 2017. Reason: errors in the materials.

**Table 4:** Pathway enrichment analysis.

	Pathway ID	Term	Genes	Bonferroni adjusted p-value	FDR
A	hsa05200	Pathways in cancer	E2F3, COL4A1, MAP2K1, MET, CDK6, WNT1, CDC42, CCND1, BCL2, VEGFA, LAMC1, AXIN2, MYC	1.93E-06	3.11E-05
	hsa04510	Focal adhesion	CDC42, CCND1, COL4A1, MAP2K1, BCL2, MET, VEGFA, COL3A1, COL1A2, LAMC1, COL1A1	2.20E-06	3.54E-05
	hsa05222	Small cell lung cancer	E2F3, CCND1, COL4A1, BCL2, CDK6, LAMC1, MYC	2.40E-04	3.90E-03
	hsa05212	Pancreatic cancer	CDC42, E2F3, CCND1, MAP2K1, VEGFA, CDK6	2.30E-04	3.20E-04
B	hsa05216	Thyroid cancer	CCND1, TP53, LEF1, MYC, TCF7L1, CTNNB1	1.28E-04	1.91E-03
	hsa04310	Wnt signaling pathway	WNT1, CCND1, CSNK1E, MMP7, TP53, LEF1, MYC, TCF7L1, CTNNB1	7.95E-04	1.19E-02
	hsa05213	Endometrial cancer	CCND1, TP53, LEF1, MYC, TCF7L1, CTNNB1	2.46E-03	3.69E-02

FDR, false discovery rate; A, pathway enrichment analysis of the verified target genes of miRNAs; B, pathway enrichment analysis of genes in the miRNAs-transcription factors-target genes network.

### Construction of an miRNA-TF-target gene network using crucial miRNAs

Totally, 353 miRNA-target gene pairs of the above 6 miRNAs (BC > 6) were predicted based on the miRecords database. Out of these target genes, E2F3, hepatic leukemia factor (HLF), lymphoid enhancer binding factor 1 (LEF1), neurofibromin 1a (NF1A), interferon regulatory factor 2 (IRF2), contactin 2 (CNTN2), E74-like factor 2 (ELF2), MYC and MYC associated factor X (MAX) were found to be TFs based on the TRANSFAC database. Using these data, a miRNA-TF-target gene network was constructed, including 5 miRNAs, 9 TFs and 55 downstream target genes of the TFs (Fig 3). miR-34a-5p, miR-34c-5p and miR-302b can regulate the target gene CCND1, Wnt family member 1 (WNT1) and MYC via the LEF1 transcription factor (Fig 3). The miR-338 was excluded from the network, because it only had one target gene, ubiquitin-conjugating enzyme E2Q family member 1 (UBE2Q1).

**Fig 3:** The miRNA-TF-target gene network. The red, yellow and green nodes represent the miRNAs, TFs and target genes of TFs, respectively. The arrows stand for regulatory relationship between two nodes. The TFs in rhombus nodes and their target genes are enriched in the Wnt signaling pathway, and the circle nodes represent the genes in uncertain signaling pathways.

Function enrichment analysis showed that the above 64 genes significantly participated in 14 GO terms (Table 3) and 3 KEGG pathways (Table 4), among which Wnt signaling pathway was the common result in these two analyses, suggesting this pathway may be of particular importance in lung cancer metastasis and curcumin treatment. Several genes, including Wnt family member 1 (WNT1), CCND1, MYC, LEF1, transcription factor 7 like 1 (TCF7L1) and catenin beta 1 (CTNNB1) were enriched, indicating they may be important therapeutic targets for lung cancer.

The article "Exploration of inhibitory mechanisms of curcumin in lung cancer metastasis using a miRNA- transcription factor-target gene network" was retracted in 2017. Reason: errors in the materials.

### PPI network

The interactions of the above 64 genes were also investigated by establishing a PPI network (Fig 4), which consisted of 31 nodes (protein) and 93 edges (PPIs). After calculating the degree of each gene (the number of edges adjacent to each node), both MYC and CCND1 were suggested to be hub genes in the PPI network, with the highest degree of 14.

**Fig 4:** PPI network. A node represents a protein, and an indirect link represents an interaction between proteins.

## Discussion

The present study identified 36 differentially expressed miRNAs between 95D cells treated with or without curcumin, 6 of which were chosen to be further investigated. By comprehensively analyzing the experimentally validated and all potential target genes of these 6 miRNAs, our study suggested miR-34a-5p, miR-34c-5p and miR-302b-3p seemed to be particularly important in inhibition of lung cancer metastasis by curcumin because their target genes (e.g. CCND1, WNT1, MYC and LEF1) were significantly enriched in metastasis related pathways (Wnt signaling pathway and Focal adhesion). As a transcription factor, LEF1 also could regulate CCND1, WNT1 and MYC. Therefore, we believe miR-34a-5p/miR-34c-5p/miR-302b-3p —LEF1—CCND1/WNT1/MYC axis may be a crucial mechanism in inhibition of lung cancer metastasis by curcumin. This conclusion seemed to be indirectly demonstrated by reviewing the literatures.

Several studies have reported that miR-34a may act as a tumor suppressor gene, with a downregulated expression in various tumor types, including lung cancer [17]. Delivery of miR-34a into cancer cells or animal models could promote cell proliferation, invasion and metastasis, which was mediated by targeted inhibition of its target genes, including CD44 [18] and MMPs (e.g. MMP9, MMP14, MMP2) [19, 20]. In addition, miR-34 was also demonstrated to regulate the TFs followed by the target genes of TFs. For example, Geng et al. confirmed miR-34a could reduce the viability and invasion of cervical cancer cells through downregulating E2F3 which then inhibited the expression of survivin [21]. Liang et al. firstly demonstrated a negative relationship between miR-34a and LEF1 expression by luciferase assays and further verified that miR-34a suppressed the migration and invasion of prostate cancer cells through increasing E-cadherin and decreasing N-cadherin in a LEF1-depedent manner [22]. In this study, we also found an important regulation relationship between miR-34a and LEF1, which has not been studied in lung cancer cells previously. Furthermore, existing evidence suggests that LEF1 is a crucial transcription factor to mediate Wnt/β-catenin signaling and participate in tumor progression [23, 24]. Thus, the expressions of Wnt signaling related genes (CCND1, WNT1 and MYC) may be regulated by LEF1 [25, 26], which was also demonstrated in our study. Also, elevated expressions of CCND1 [27], WNT1 [28] and MYC [29] were shown to be associated with malignant characters of lung cancer, leading to an unfavorable prognosis. Accordingly, we have reasons to trust that miR-34a (downregulated)—LEF1 (upregulated)—CCND1/WNT1/MYC (upregulated) axis may be an important target for inhibition of lung cancer metastasis and to upregulate miR-34a may be an underlying strategy to achieve this goal. As expected, our study showed miR-34a was significantly upregulated by curcumin (FC = 7.26), which was in line with previous studies in other cancers [30, 31].

miR-302b also seems to be a potential molecular marker for cancer invasion and metastasis [32]. miR-302b is downregulated in hepatocellular carcinoma cancer specimens and overexpression of miR-302b suppresses invasion and metastasis by directly targeting AKT2 followed by regulation of NF-κB and MMP-2 in human hepatocellular carcinoma cells [33]. Similarly, miR-302b was found to be significantly lowly expressed in high-metastatic lung cancer cell line 95D than that in low metastatic cell line 95C. Transfection of miR-302b exerts anti-proliferation and anti-migration effects on 95D cells, which was accompanied with significantly down-regulated expression of TGFβRII, phosphorylated ERK1/2 and MMP9 induced by TGF-β1 [34]. However, the inhibitory mechanism of miR-302b on cancer remains unclear and its regulation on transcription factor is rarely reported [35]. In this study, we first found miR-302b might be involved in lung cancer metastasis by regulating LEF1 followed by Wnt signaling related genes, which need a further experiment confirmation. Although growing evidence has indicated that upregulation of miR-302b may be an important mechanism during cancer treatments [36], whether the expression of miR-302b can be changed after curcumin seems not to be investigated. We first demonstrated miR-302b was significantly upregulated (FC = 3.34) when treatment with 10 μM curcumin, which also needs a further experiment confirmation.

The article "Exploration of inhibitory mechanisms of curcumin in lung cancer metastasis using a miRNA- transcription factor-target gene network" was retracted in 2017. Reason: errors in the materials.

As a member of miR-34 conserved family, miR-34c plays a similar role with miR-34a theoretically. However, in our study, we found miR-34c was significantly downregulated (FC = 0.37) after treatment with 10 μM curcumin, indicating miR-34c may be a proto-oncogene. This conclusion seemed to be supported by a recent study which indicated forced expression of miR-34c may contribute to resistance to caspase-8-induced apoptosis in lung cancer cells [37]. Nevertheless, it is essential to further explore how miR-34c, miR-34a and miR-302b collectively to regulate LEF1 followed by Wnt signaling related genes in lung cancer [38].

Although a great amount of documentary evidence has indicated its anti-carcinogenesis properties, extensively bringing curcumin to the clinic remains a difficult process because of poor oral bioavailability due to low absorption [39]. Recently, scholars have attempted to encapsulate or incorporate curcumin in nanoparticles to enhance curcumin delivery [39]. As expected, concentration of curcumin was increased in mice via *i*.*p*. after loaded with solid lipid nanoparticles (SLN). Furthermore, SLN-curcumin enhanced the targeting of curcumin to lung and tumor, finally improving the inhibition efficiency of curcumin to 69.3% from 19.5% [40]. However, other strategies [(such combination of curcumin and its target miRNAs (miR-34a and miR-302b) mimics)] to enhance the therapeutic effects are needed to be further investigated.

## Conclusions

Our present study provides some novel, underlying mechanisms of curcumin (miR-34a-5p/miR-34c-5p/miR-302b-3p— LEF1—CCND1/WNT1/MYC axis) on lung cancer metastasis. Further *in vitro* and *in vivo* experimental studies were necessary to confirm these findings and explore combination strategies to enhance the therapeutic efficiency of curcumin.
